# ACEI and ARB Lower the Incidence of End-Stage Renal Disease among Patients with Diabetic Nephropathy: A Meta-analysis

**DOI:** 10.1155/2022/6962654

**Published:** 2022-05-31

**Authors:** Xiaojuan Deng, Dayun Li, Qiufeng Tang, Yueyao Chen

**Affiliations:** ^1^Department of Pharmacy, Geriatric Hospital of Hainan, Haikou, 571100 Hainan, China; ^2^Department of Pharmacy, Ling Shui Li Autonomous County People's Hospital, Lingshui, 572400 Hainan, China; ^3^Department of Nephrology, DanZhou People's Hospital, Danzhou, 571700 Hainan, China

## Abstract

**Objective:**

This study explores the effects of Angiotensin-Converting Enzyme Inhibitors (ACEI) or Angiotensin Receptor Blockers (ARB) on the incidence of end-stage renal disease (ESRD) in diabetic nephropathy (DN) patients.

**Methods:**

Literatures were searched in PubMed, Embase, Medline, CENTRAL, and CNKI databases. These literatures included a randomized controlled trial to evaluate the efficacy of ACEI and ARB among patients with DN. The endpoint event included the occurrence of ERSD. Risk ratio (RR) and 95% confidence interval (CI) were used to represent the combined effect size. A fixed-effect model was used to analyze if heterogeneity did not exist between literatures. If heterogeneity exists between literatures, a random-effect model was used to analyze. The source of heterogeneity was explored by subgroup analysis and sensitivity analysis.

**Results:**

A total of 11 literatures were included in the study. The RR of ESRD was 0.79 (95% CI (0.79, 0.90), *Z* = 3.58, *P* = 0.0003) in the patients treated with RAS blockers compared with placebo, and there was no heterogeneity between studies (Chi^2^ = 5.09, *P* = 0.88, *I*^2^ = 0%). The funnel plot showed that the scatter point was biased to the left with publication bias. The RR of ESRD was 0.63 (95% CI (0.41, 0.95), *Z* = 2.18, *P* = 0.03) in the patients treated with ACEI compared with placebo. There was no heterogeneity between studies (Chi^2^ = 2.23, *P* = 0.95, *I*^2^ = 0%). Compared with placebo, RR of ESRD among patients with ARB intervention was 0.81 (95% CI (0.71, 0.93), *Z* = 3.00, *P* = 0.003). There was no heterogeneity between studies (Chi^2^ = 1.49, *P* = 0.48, *I*^2^ = 0%).

**Conclusion:**

ACEI and ARB can reduce the risk of ESRD among diabetic nephropathy patients.

## 1. Introduction

In recent years, the incidence of diabetes mellitus, primarily type 2 diabetes, gradually increased [1–3]. Diabetic nephropathy (DN) is one of the most common complications of diabetes [4, 5]. The end-stage renal disease (ESRD) is irreversible, which often diagnosed in the advanced stage [4]. DN is the most common single cause of ESRD [5]. The proportion of ESRD caused by diabetic nephropathy is increasing, which may be related to the increase in the diabetes incidence rate and the prolongation of the life span of diabetic patients [5]. Patients with diabetic nephropathy need to maintain dialysis or receive kidney transplantation [6, 7]. These treatment methods bring heavy economic and psychological burdens and occupy a lot of medical resources [7]. Delaying the progression of DN has important clinical significance [7].

For diabetic patients, the role of renin-angiotensin system (RAS) blockers, including Angiotensin-Converting Enzyme Inhibitors (ACEI) and Angiotensin Receptor Blockers (ARB), has been controversial in improving clinical prognosis and reducing clinical events. According to a meta-analysis, ACEI and ARB have the advantage of [8] in treating diabetic nephropathy compared with other antihypertensive drugs. However, meta-analysis studies indicated that ACEI and ARB in reducing the risk of kidney events in diabetic patients are not superior to other antihypertensive drugs [9]. In diabetic nephropathy, a randomized controlled study showed that although ACEI could reduce the risk of serum creatinine double the baseline, it did not affect the incidence of ESRD ([10]). Therefore, a meta-analysis helps explore whether ACEI and ARB drugs can reduce the incidence of ESRD among patients with DN.

## 2. Materials and Methods

### 2.1. Literature Retrieve

Literature search was performed in MEDLINE, PubMed, Embase, CENTRAL, and CNKI databases. The search terms were ((“ACEI” OR “ARB” OR “RAS” OR “Angiotensin-Converting Enzyme Inhibitors” OR “Angiotensin Receptor Blockers” OR “Renin angiotensin system”) AND (“diabetes” OR “diabetic nephropathy”). There are no restrictions on literature language, publication time, and follow-up duration.

### 2.2. Literature Screening

Literature included the following criteria: (1) subjects were diabetic nephropathy patients; (2) the experimental group and control group were set up. The experimental group was treated with ACEI drugs or ARB drugs. The control group was treated with placebo; (3) endpoint events included the occurrence of terminal nephropathy; and (4) randomized controlled study.

Exclusion criteria are as follows: (1) repeated reports, (2) the balance of baseline data was poor, (3) the experimental group was treated with other drugs besides ACEI drugs, and (4) the literature data was missing and cannot be supplemented.

### 2.3. Data Extraction

In this paper, two researchers jointly extracted the author, title, publication time, number of researchers in the control and experimental groups, number of patients with ESRD, etc. For the data that could not be obtained in the literature, the researchers contacted the author to obtain it. If two researchers disagree on the data, an agreement was achieved through discussion.

### 2.4. Literature Quality Evaluation

In this paper, two researchers applied the Jadad scale to evaluate the quality of the included RCT research, including the generation method of random sequence, randomized hiding, the use of blind method, withdrawal, and withdrawal rules.

### 2.5. Heterogeneity Test and Publication Bias Test

Chi-square test was applied for the heterogeneity test. If *I*^2^ > 50% or *P* < 0.1, it was considered that there was heterogeneity among published literatures, and a random effect model was used. In order to show the causes of heterogeneity, subgroup analysis and sensitivity analysis were conducted. If *I*^2^ ≤ 50% and *P* ≥ 0.1, it was considered that no heterogeneity was among the published literatures, and the fixed effect model was used. Publication bias test was conducted by funnel plot.

### 2.6. Statistical Method

This study used the Cochrane software RevMan5.3 statistical analysis of the data. Risk ratio (RR) value and 95% confidence interval (CI) were calculated using Mantel-Haenszel statistical method. Bilateral *P* < 0.05 indicated statistically significant.

## 3. Results

### 3.1. Characteristics of Included Literature

A total of 2486 literatures were retrieved in the above database. A total of 2475 literatures were excluded, with 11 literatures included in the study [10–20]. The flow chart of literature screening is shown in Figure 1. The basic information of literature and the Jadad score are shown in Table 1.

### 3.2. RAS Blockers Reduce the Incidence of ESRD

A total of 11 articles were included, including 7595 diabetic nephropathy patients. 337 of 3793 patients in the RAS blocker drug intervention group had ESRD. As shown in Figure 2, 423 of the 3802 people in the placebo control group developed the ESRD. The heterogeneity test showed that no heterogeneity was among the studies (Chi^2^ = 5.09, *P* = 0.88, *I*^2^ = 0%). The combined analysis showed that the RR of patients with ESRD treated with RAS blocker was 0.79 compared with placebo (95% CI (0.79, 0.90), *Z* = 3.58, *P* = 0.0003). As shown in Figure 3, the funnel plot demonstrated that the scatter points were biased to the left, and there was publication bias.

### 3.3. ACEI and ARB Reduce the Incidence of ESRD

Subgroup analysis was carried out according to different drugs, divided into ACEI and ARB subgroups. Eight literatures were included in the ACEI subgroup. The heterogeneity test showed that no heterogeneity was among the studies (Chi^2^ = 2.23, *P* = 0.95, *I*^2^ = 0%). The combined analysis showed that compared with placebo, the RR of patients with end-stage renal disease after ACEI intervention was 0.63 (95% CI [0.41, 0.95], *Z* = 2.18, *P* = 0.03) as shown in Figure 4. Three articles were included in the ARB subgroup. Heterogeneity test showed that no heterogeneity was among the studies (Chi^2^ = 1.49, *P* = 0.48, *I*^2^ = 0%). The combined analysis showed that compared with placebo, the RR of patients with end-stage renal disease after ARB intervention was 0.81 (95% CI (0.71, 0.93), *Z* = 3.00, *P* = 0.003) as shown in Figure 4.

## 4. Discussion

A total of 11 literatures were included in this study for meta-analysis with no heterogeneity among the literatures. Meta-analysis showed that renin-angiotensin system blocker could reduce the incidence of ESRD among patients with DN. The angiotensin and ACEI subtypes were divided into two groups. NO heterogeneity was among studies in ACEI subgroups, such as ARB subgroups. Meta-analysis of the ACEI and ARB subgroups showed that ACEI and ARB drugs could reduce the risk of ESRD among patients with DN. The results of the subgroup analysis were consistent with the overall analysis. A previous meta-analysis [21] showed that ACEI treatment did not affect the renal outcome, while ARB treatment significantly reduced the risk of ESRD. We believe that the conclusions of this study are controversial. The study conducted a sensitivity analysis, excluding the study of Patel [22], and concluded that ACEI drugs could reduce the incidence of ESRD. Unfortunately, they did not conclude with the results of the sensitivity analysis. We also looked at Patel et al.'s findings for diabetes patients, not diabetic nephropathy patients, and combined ACEI and diuretics. Therefore, it was not included in our study. In addition, we also noted a randomized controlled study [23], showing that ACEI drugs could reduce the risk of DN and the risk of cardiovascular adverse events. Class ACEI drugs can protect cardiovascular and kidneys in diabetic patients. However, we cannot get the full text because the study was aimed at diabetic patients, not diabetic nephropathy patients. The information in the summary section could not provide the data information needed in this study because this randomized study had not been included in our analysis.

At present, meta-analysis of ACEI and ARB has little effect on renal protection among patients with DN. Some meta-analyses explored the effects of the two drugs on the kidney of diabetic patients [8, 9, 24]. A meta-analysis [8], which included 28 RCT trials, found that ACEI and ARB drugs had protective effects on the kidney among patients with type 2 diabetes compared with other antihypertensive drugs and placebo. Another meta-analysis of [24] included 63 RCT trials, including 36917 diabetic patients. The results showed that ACEI drugs had renal protective effects on diabetic patients, while ARB drugs did not show their protective effects on the kidneys. Another meta-analysis of 19 RCT studies [9] showed that ACEI and ARB were not superior to other antihypertensive drugs in reducing all-cause death, cardiovascular time, and renal events. These meta-analyses obtained inconsistent conclusions, which may be related to the differences in research objects, the differences in intervention schemes in the control group, and the different definitions of endpoint events. There was heterogeneity in clinical manifestations of diabetes, including prognosis.

There are also some limitations in our research. First of all, we did not distinguish between type 1 diabetes and type 2 diabetes. There are differences in the pathogenesis of type 1 diabetes and type 2 diabetes and differences in the course of the disease, clinical manifestations, prognosis, and sensitivity to drugs, which may impact our results. Further studies are needed to confirm whether there is a difference in efficacy between RAS inhibitors in type 1 and type 2 diabetes. Secondly, our study did not distinguish the effects of different doses of ACEI and ARB on diabetic nephropathy. Previous studies have shown that these two drugs slow down the decline of albuminuria and glomerular filtration rate in a dose-dependent manner [20]. Thirdly, we did not explore the efficacy of RAS inhibitors in diabetes patients of different ages, genders, and diets. All of these clinical variables may influence outcomes. Finally, most of the research data we obtained came from developed countries, which may also bias our results.

In particular, some studies have pointed out that the combination of ARB and ACEI drugs may lead to hyperkalemia and increase the risk of acute renal injury [25]. However, this study concluded that ACEI and ARB drugs have protective effects on the kidney among patients with diabetic nephropathy. However, it is still necessary to conduct a large-scale RCT study with multiple centers to observe the effectiveness and safety of different doses and drug regimens.

In summary, this study suggests that ACEI and ARB drugs can reduce the risk of ESRD among patients with DN.

## Figures and Tables

**Figure 1:** Document screening flow chart.

**Figure 2:** Forest diagram of the effect of RAS blocker and placebo on the incidence of end-stage renal disease.

**Figure 3:** Funnel plot of the effect of RAS blocker and placebo on the incidence of end-stage renal disease. OR stands for odd ratio; SE stands for standard error.

**Figure 4:** Forest map of the effects of ACEI and ARB versus placebo on the incidence of end-stage renal disease.

**Table 1:** Literature characteristics and Jadad score.

Study and year	No. of ESRD	No. of patients	Diabetes type	Jadad
Bauer [11], 1992	3	33	Mixed	3
Brenner [16], 2001	341	1513	2	4
Imai [15], 2011	153	586	2	5
Katayama [14], 2002	6	79	1	5
Lewis [18], 1993	36	409	1	5
Lewis [17], 2001	183	1149	2	4
Marre [10], 2004	14	3627	2	3
Maschio [19], 1996	7	21	2	5
Parving [20], 1989	5	32	1	3
Ravid [12], 1993	9	108	2	5
Tong [13], 2006	3	38	2	4

## Data Availability

The data used to support the findings of this study are included within the article.
